# Genetic Association of ERCC6 rs2228526 Polymorphism with the Risk of Cancer: Evidence from a Meta-Analysis

**DOI:** 10.1155/2022/2662666

**Published:** 2022-04-15

**Authors:** Xiaochun Lin, Yongfu Wu, Qingde Li, Hongying Yu, Xugui Li, Xiaohua Li, Jinkun Zheng

**Affiliations:** Department of Pharmacy, Yuebei People's Hospital, Shaoguan, Guangdong, China

## Abstract

At present, several studies have assessed the association between ERCC6 rs2228526 polymorphism and the risk of cancer. However, the association remained controversial. To provide a more accurate estimate on the association, we performed a meta-analysis search of case-control studies on the associations of ERCC6 rs2228526 with susceptibility to cancer. PubMed, Embase, Google Scholar, Wanfang database, and Chinese National Knowledge Infrastructure databases (CNKI) China Biological Medicine Database (CBM) (up to August 2021) were searched to identify eligible studies. The effect summary odds ratio (OR) with 95% confidence intervals (CI) was applied to assay the association between the ERCC6 rs2228526 polymorphism and the risk of cancer. 14 studies included 15 case-control studies which contained 5,856 cases, and 6,387 controls were finally determined as qualified studies for this meta-analysis. Overall, based on current studies, we found significant association between ERCC6 rs2228526 polymorphism and the risk of cancer in four genetic models [the allele model G vs. A: 1.10, (1.03–1.17); the homozygous model GG vs. AA: 1.27, (1.07–1.51); heterozygote model GA vs. AA: 1.08, (1.00–1.17); the dominant model GG + GA vs. AA: 1.10, (1.02–1.19); the recessive model GG vs. GA + AA: 1.22, (1.03–1.45)]. In the stratified analysis based on ethnicity, we found significant association in two genetic models in Asians. Further, significant genetic cancer susceptibility was found under PB control on subgroup analysis by source of control. In addition, no significant association was found in lung cancer and bladder cancer patients in subgroup analyses based on cancer style. This study suggests that the ERCC6 rs2228526 polymorphism may be associated with increased cancer risk.

## 1. Introduction

The report from the GLOBOCAN 2020 from WHO showed that there were 10 million cancer deaths (9.9 million nonmelanoma skin cancer were excluded) and 19.3 million new cancer cases (18.1 million nonmelanoma skin cancer were excluded) in 2020 [1]. Cancer is a complex disease, the exact mechanism of carcinogenesis is still not clear. An increasing number of studies have showed that the occurrence of cancer may be influenced by both genetic factors and environmental [2, 3]. In addition, many genes have been identified as cancer-susceptible genes.

The pathway of nucleotide-excision repair (NER) involved the DNA repair pathway which could repair different lesions in DNA [4, 5]. The DNA repair capacity may change and consequently contribute to the development of carcinogenesis when the genetic variant in this pathway is related to gene. [6]. The gene of excision repair cross-complementing group 6 (ERCC6), also known as Cockayne syndrome group B (CSB),which is located on human chromosome 10q11, is an important component of the NER pathway which participates in base excision DNA repair. Single nucleotide polymorphisms have been identified in several exons of the ERCC6 gene, such as rs2228528, rs228526, and rs2228529. The mutant of ERCC6 gene has been largely investigated in a variety of cancers [7–9], but the effect of ERCC polymorphism in different genetic loci and cancers is not same.

One common G/A polymorphism in its coding region is ERCC6 rs2228526 which can result in an amino acid alteration within the protein sequence for a methionine change to valine transition in codon 1097 (Met1097Val) [10]. This mutation in the ERCC6 rs2228526 may diminish its activity, further resulting in a defect in overall NER pathway. Recent studies have reported the association between ERCC6 rs2228526 polymorphism and risks of various cancers [7, 10–22]. However, the results of these studies remained controversial. To provide a more accurate estimate on the association, we performed a meta-analysis to assess whether ERCC6 rs2228526 polymorphism increases the risk of cancer.

## 2. Materials and Methods

### 2.1. The Literature Search Strategy

PubMed, Embase, Google Scholar, Wanfang database, and Chinese National Knowledge Infrastructure databases (CNKI) China Biological Medicine Database (CBM) (up to August 2021) were searched to identify eligible studies. The structured strategies used the following search terms: “ERCC6”, “CSB”, “rs2228526”, “polymorphism”, “cancer”, and “carcinoma”. In addition, the reference lists of identified studies were manually checked to include other potentially eligible trials. A manual search of bibliographies of identified studies was also performed for other relevant eligible publications.

### 2.2. Inclusion and Exclusion Criteria

The inclusion criteria of these eligible studies in the meta-analysis were as follows: The study was designed as a case control and contained cancer genotyping. The exclusion criteria were as follows: duplicate of earlier publication and no usable genotype frequency data.

### 2.3. Data Extraction

Two authors (Xiaochuan Lin and Yongfu Wu) independently extracted and cross-checked the data from eligible studies. For each study, the information was collected as follows: year of publication, first author, region, ethnicity, cancer type, number of genotype controls and cases, and genotype frequency, respectively. The different races are divided into Asian, Caucasian, and African-Americans. Further discussions among all authors were performed to resolve the disagreements.

### 2.4. Statistical Analysis

The effect summary odds ratio (OR) with 95% confidence intervals (CI) was applied to assay the association between the ERCC6 rs2228527 polymorphism and the risk of cancer in this meta-analysis. We used the Hardy–Weinberg equilibrium (HWE) to test the equilibrium in the controls, and it would consider significant disequilibrium when *p* < 0.05. The significance of pooled ORs was assessed by *Z*-test. The heterogeneity of the studies was assessed by *χ*^2^-based Q statistical test. If *I*^2^ > 50% and *P*_*Q*_ < 0.10, the pooled OR was calculated by the random-effects model. Otherwise, the fixed-effects mode was used. The allelic model (*G vs. A*), homozygous model (*GG vs. AA*), heterozygote model (*GA vs. AA*), dominant model (*GG + GA vs. AA*), and recessive model (*GG vs. GA + AA*) genetic models were performed, respectively. We also perform subgroup analysis based on ethnicity, cancer style, source of control, and genotyping method. Sensitivity analysis was used to assess the stability of the results. Publication bias was detected by funnel plot and estimated Egger's tests. The STATA software (version 12.0) was used for data analysis.

#### 2.4.1. Trial Sequential Analysis (TSA)

The TSA software (version 0.9.5.10 Beta) was used to perform the trial sequential analysis. Our study sets the overall 5% risk of a type I error and 20% risk of a type II error (power of 80%) to evaluate the required information size (RIS). In TSA, if the cumulative *Z* value crosses the RIS threshold or the required information size has been reached, it can be considered the sample size of the accumulated evidence is sufficient. However, if the cumulative *Z* value does not cross the RIS threshold, it means the sample size is not sufficient. And it still needs more studies to confirm the results [23, 24].

## 3. Results

### 3.1. Identification of Eligible Studies

Based on the inclusion and exclusion criteria, 512 potentially relevant studies were retrieved by the initial database search in PubMed, Embase, Google Scholar, Wanfang database, and Chinese National Knowledge Infrastructure databases (CNKI) China Biological Medicine Database (CBM). 456 studies were excluded because they were not associated with ERCC RS2228526 polymorphism. An additional 456 studies were excluded for the following reasons: 67 repeated studies and 361 unrelated studies, 28 meta-analysis and review. In addition, further 43 studies were not included due to the following: 33 not related to ERCC rs2228526 and 9 not case-control studies. Finally, 14 studies included 15 case-control studies which contained 5,856 cases, and 6,387 controls were finally determined as qualified studies for this meta-analysis. The detailed process of excluding and selecting studies is shown in Figure 1.

### 3.2. Characteristics of Published Studies

Fourteen studies contain fifteen case-control studies published in English until 2019 were identified eligible studies in this meta-analysis. The detailed characteristics of these studies are shown in Table 1. Five of the included studies were from China, seven from the United States, one from Spain, and two from Belarus. The genotype distributions of the control groups in each studies conform to the HWE equilibrium except two (*p* > 0.05) (Table 1). This meta-analysis also included studies with controls that did not conform to HWE, but these studies were excluded when we assess the stability of the results.

### 3.3. Meta-Analysis Results

Overall, this meta-analysis results suggest that ERCC rs2228526 polymorphism was significantly associated with genetic susceptibility of cancer [the allele model G vs. A: 1.10, (1.03–1.17); the homozygous model GG vs. AA: 1.27, (1.07–1.51); heterozygote model GA vs. AA: 1.08, (1.00–1.17); the dominant model GG + GA vs. AA: 1.10, (1.02–1.19); and the recessive model GG vs. GA + AA: 1.22, (1.03–1.45);, respectively] (Figures 2–6). When the genotype distribution of these studies in the control group deviated from HWE were excluded, the meta-analysis results were not significantly changed. Subgroup analysis by cancer style suggested that there were no significant associations which were observed among lung and bladder cancer under all genetic models. However, in the stratified analysis based on ethnicity, we found significant association in two genetic models in Asians (Table 2). In addition, when subgroup analysis was performed by control source, hospital-based controls also showed significant differences (Table 2).

### 3.4. Sensitivity Analysis

Sensitivity analysis was used to verify that whether pooled results were changed when one of these studies was removed. When one of the studies was deleted (data not shown), the pooled OR and 95% CI did not change significantly, suggesting that any single study had little impact on the overall OR.

### 3.5. Publication Bias

Egger's linear regression test and Begg's funnel plot were used to assay the publication bias of this study. No evidence of publication bias was detected by both Egger's and Begg's test (Table 3).

### 3.6. Trial Sequential Analysis Results

The TSA was conducted in the homozygous model (GG vs. AA). The result showed that the cumulative *Z*-curve (blue line) had crossed the TSA boundary (red straight lines) and the sample size had reached the required information sizes (*n* = 6874) (Figure 7). These data indicated that the cumulative evidence on the ERCC6 rs2228526 polymorphism was adequate.

## 4. Discussion

The pathogenesis of cancer is complex, it is mainly related to the multifactorial of genetic susceptibility and environmental factors [25]. It is known that the nucleotide excision repair (NER) pathway is thought to modulate DNA repair, and abnormalities in this pathway may be associated with the risk of cancer [26]. Excision repair cross-complementing group 6 (ERCC6) gene is an important component of the NER pathway which participates in base excision DNA repair [13]. The polymorphism in the ERCC6 gene may affect DNA repair ability in the general population and lead to genetic susceptibility to cancer [22]. Recently, due to the ERCC6 gene played an important role of in the NER pathway, the ERCC6 RS2228526 polymorphism has been studied in a variety of cancers. However, the results of these studies are inconsistent due to small sample sizes and different populations. Gu et al. revealed that the G allele of codon 1097 is associated with better DNA repair capacity [27]. Chang et al. suggest a significantly different distribution was not found in the frequency of the ERCC6 codon 1097 between the bladder cancer and control groups [10]. Ma et al. found that ERCC6 rs2228526 polymorphism was associated with a significantly increased lung cancer risk [13]. Chiu et al. showed that a different distribution was also not found in the frequency of the ERCC6 codon 1097 between the oral cancer and control groups [11]. In order to obtain a more accurate association estimate, we conducted a meta-analysis to find the association between ERCC6 rs2228526 polymorphism and the risk of cancer.

In this meta-analysis, 14 literatures included 15 case-control studies which contained 5,856 cases, and 6,387 controls were finally determined as qualified studies for this meta-analysis. The HWE test results showed that, except for one study reported by Rajaraman et al., the genotypic distributions of all eligible studies in the control group are consistent with the HWE equilibrium [14]. This meta-analysis showed a significant association between ERCC6 rs2228526 polymorphism and cancer susceptibility. When the study which is not consistent with the HWE equilibrium was excluded from this meta-analysis, this association between ERCC6 rs2228526 polymorphism and cancer risk was not alerted. In addition, the sensitivity analysis results indicated that when we excluded one of these studies, the combined OR was not significantly alerted. Besides, the heterogeneity was not significantly found and TSA result indicated that the cumulative evidence on the ERCC6 rs2228526 polymorphism was adequate which suggested our findings were more robust. Furthermore, in the stratified analysis based on ethnicity, we found significant association in two genetic models in Asians but no significant difference was found in other ethnicity. Further, significant associations were found under PB control in subgroup analyses based on source of control. In addition, no significant association was found in lung cancer and bladder cancer patients in subgroup analyses based on cancer style.

It should be noted that this study has some limitations. Firstly, owing to the limited data, we did not perform a subgroup analysis of other factors that may be involved in the disease progression, such as age, smoking, and other lifestyles. Secondly, in the subgroup analysis, the sample sizes of controls and cases were not large. Thirdly, we just used the unadjusted data to assess the association between ERCC6 rs2228526 polymorphism and cancer risk in this meta-analysis. It is hard to gain more precise conclusions. Finally, it may lead to biased results for the searches in this meta-analysis which is just limited in the Chinese and English study. To sum up, our findings should be cautiously interpreted on account of abovementioned limitations.

In summary, this meta-analysis demonstrated the there was a significant association between ERCC6 rs2228526 polymorphism and cancer risk according to the current published literatures. However, further researches with well-designed and large samples are needed to validate these results. Besides, further studies with gene–environment interactions and gene–gene are needed to give more reliable results for this association.

## Figures and Tables

**Figure 1:** Flowchart of the process used for selection of eligible studies.

**Figure 2:** Forest plot of the meta-analysis on the association between ERCC6 rs2228526 polymorphism and cancer risk in allele model (G vs. A). Error bars indicate 95% CI. Solid squares represent each study in the meta-analysis. Solid diamonds represent pooled OR.

**Figure 3:** Forest plot of the meta-analysis on the association between ERCC6 rs2228526 polymorphism and cancer risk in homozygous model (GG vs. AA). Error bars indicate 95% CI. Solid squares represent each study in the meta-analysis. Solid diamonds represent pooled OR.

**Figure 4:** Forest plot of the meta-analysis on the association between ERCC6 rs2228526 polymorphism and cancer risk in heterozygote model (GA vs. AA). Error bars indicate 95% CI. Solid squares represent each study in the meta-analysis. Solid diamonds represent pooled OR.

**Figure 5:** Forest plot of the meta-analysis on the association between ERCC6 rs2228526 polymorphism and cancer risk in dominant model (GG + GA vs. AA). Error bars indicate 95% CI. Solid squares represent each study in the meta-analysis. Solid diamonds represent pooled OR.

**Figure 6:** Forest plot of the meta-analysis on the association between ERCC6 rs2228526 polymorphism and cancer risk in recessive model (GG vs. GA + AA). Error bars indicate 95% CI. Solid squares represent each study in the meta-analysis. Solid diamonds represent pooled OR.

**Figure 7:** Trial sequential analysis of the association between ERCC6 rs2228526 polymorphism and cancer risk in homozygous model (GG vs. AA).

**Table 1:** Association between individual study characteristics and ERCC6 rs2228526 polymorphism.

Reference	Year	Area	Ethnicity	Cancer style	Source of control	Cases	Controls	Cases			Controls			HWE (control)	Genotyping
								AA	AG	GG	AA	AG	GG	*p*	Method
Chang et al.	2009	China	Asian	Bladder cancer	HB	288	288	248	36	4	242	43	3	0.443	PCR-RFLP
Chiu et al.	2008	China	Asian	Oral cancer	HB	292	290	259	30	3	243	44	3	0.455	PCR-RFLP
Huang et al.	2006	America	Mix	Colorectal adenoma	HB	646	657	405	211	30	410	224	23	0.284	National Cancer Institute Core Genotyping Facility
Ma et al.	2009	China	Asian	Lung cancer	PB	500	504	429	69	2	451	51	2	0.653	Illumina SNP genotyping BeadLab platform
Rajaraman et al.	2008	America	Mix	Breast cancer	HB	790	1070	510	241	39	704	312	54	0.015	TaqMan
Ramaniuk et al.	2014	Belarus	Caucasian	Bladder cancer	PB	336	369	167	145	24	187	152	30	1.000	PCR-RFLP
Zhang et al.	2014	China	Asian	Prostate cancer	HB	229	238	90	105	34	113	103	22	0.880	MassARRAY platform
Zheng et al.	2010	America	Caucasian	Lung cancer	HB and PB	161	281	97	55	9	170	95	16	0.744	TaqMan
Zheng et al.	2010	America	African Americans	Lung cancer	HB and PB	59	175	43	14	2	130	40	5	0.528	TaqMan
Ibarrola-Villava et al.	2011	Spanish	Caucasian	Malignant melanoma	HB	684	406	339	215	30	253	137	16	0.763	TaqMan
Pan et al.	2009	America	Caucasian	Esophageal cancer	HB	382	452	235	125	22	291	147	14	0.452	TaqMan
Wu et al.	2006	America	Caucasian	Bladder cancer	HB	605	595	371	204	30	392	182	21	1.000	TaqMan
Yang et al.	2013	China	Asian	Prostate cancer	HB	229	238	90	105	34	113	103	22	0.881	PCR-RFLP
Savina et al.	2017	Belarus	Caucasian	Bladder cancer	PB	419	354	207	182	30	176	148	30	1.000	PCR-RFLP
Han et al.	2008	America	Mix	Breast cancer	PB	236	470	134	89	13	288	161	21		Illumina high-multiplex BeadArray genotyping system

Abbreviations: HB = hospital based; PB = population based; HWE = Hardy–Weinberg equilibrium; F = fixed-effects mode; R = random-effects model.

**Table 2:** Main results of pooled ORs in the meta-analysis.

Study groups	No. of study	Sample size (cases/controls)	G vs. A			GG vs. AA			GA vs. AA			GA + GG vs. AA			GG vs. GA + AA		
			OR [95% CI]	*I* ^2^ (%)	Model	OR [95% CI]	*I* ^2^ (%)	Model	OR [95% CI]	*I* ^2^ (%)	Model	OR [95% CI]	*I* ^2^ (%)	Model	OR [95% CI]	*I* ^2^ (%)	Model
Overall	15	5856/6837	1.10 [1.03, 1.17]	11.7	F	1.27 [1.07, 1.51]	0	F	1.08 [1.00, 1.17]	0	F	1.10 [1.02, 1.19]	0	F	1.22 [1.03, 1.45]	0	F
Cancer style																	
Bladder cancer	4	1648/1606	1.05 [0.93, 1.18]	0	F	1.05 [0.77, 1.44]	0	F	1.08 [0.92, 1.25]	0	F	1.07 [0.93, 1.24]	0	F	1.01 [0.74, 1.38]	0	F
Lung caner	3	720/960	1.14 [0.91, 1.43]	0	F	1.00 [0.55, 1.83]	0	F	1.19 [0.92, 1.55]	0	F	1.18 [0.92, 1.52]	0	F	1.00 [0.55, 1.82]	0	F
Prostate cancer	2	458/476	1.361.12, 1.65]	0	F	1.07 [0.74, 1.55]	0	F	1.10 [0.92, 1.31]	0	F	1.09 [0.93, 1.29]	0	F	1.02 [0.50, 2.05]	0	F
Breast cancer	2	1026/1540	1.07 [0.93, 1.23]	0	F	1.94 [1.27, 2.97]	0	F	1.28 [0.97, 1.68]	0	F	1.40 [1.08, 1.81]	0	F	1.71 [1.14, 2.56]	0	F
Other cancer	4	2004/1805	1.08 [0.96, 1.21]	41.5	F	1.46 [1.03, 2.07]	0	F	1.00 [0.87, 1.16]	36.4	F	1.04 [0.91, 1.20]	41.7	F	1.44 [1.02, 2.04]	0	F
Ethnicity																	
Asian	5	1538/1558	1.14 [0.90, 1.45]	59	R	1.77 [1.20, 2.61]	0	F	1.07 [0.81, 1.42]	55.3	R	1.12 [0.84 1.50]	60.4	R	1.61 [1.11, 2.23]	0	F
Caucasian	6	2587/2457	1.10 [1.00, 1.21]	0	F	1.19 [0.92, 1.53]	8	F	1.10 [0.98, 1.24]	0	F	1.12 [1.00, 1.25]	0	F	1.14 [0.89, 1.46]	7.3	F
African Americans	1	59/175	1.08 [0.60, 1.94]	—	—	1.21 [0.23, 6.46]	—	—	1.06 [0.53, 2.13]	—	—	1.07 [0.55, 2.09]	—	—	1.19 [0.23, 6,32]	0	F
Mix	3	1672/2197	1.06 [0.94, 1.18]	0	F	1.14 [0.84, 1.55]	0	F	1.04 [0.91, 1.20]	0	F	1.03 [0.92, 1.21]	0	F	1.12 [0.83, 1.52]		
Source of controls																	
HB	9	4145/4234	1.16 [1.06, 1.27]	31.6	F	1.49 [1.17, 1.90]	0	F	1.12 [1.00, 1.25]	16.1	F	1.16 [1.04, 1.29]	26.5	F	1.40 [1.11, 1.77]	0	F
PB	4	1491/1697	1.04 [0.94, 1.15]	0	F	1.06 [0.81, 1.39]	0	F	1.04 [0.92, 1.18]	0	F	1.05 [0.93, 1.18]	0	F	1.14 [0.80, 1.36]	0	F
HB, PB	2	220/456	1.02 [0.77, 1.36]	0	F	1.03 [0.48, 2.20]	0	F	1.03 [0.72, 1.47]	0	F	1.03 [0.73, 1.44]	0	F	1.02 [0.48, 2.16]	0	F
Genotyping method																	
PCR-RFLP	5	1564/1539	1.02 [0.90, 1.15]	48.1	F	1.11 [0.81, 1.52]	17.1	F	1.00 [0.85, 1.18]	28.9	F	1.01 [0.86, 1.18]	39.7	F	0.92 [0.56, 1.52]	2.5	F
TaqMan	6	2681/2979	1.12 [1.02, 1.23]	0	F	1.27 [0.98, 1.64]	0	F	1.10 [0.98, 1.24]	0	F	1.12 [1.01, 1.26]	0	F	1.23 [0.95, 1.58]	0	F
Other methods	4	1611/1869	1.16 [1.03, 1.32]	18.7	F	1.50 [1.06, 2.13]	0	F	1.12 [0.96, 1.31]	22.8	F	1.16 [1.00, 1.35]	25.1	F	1.431.02, 2.01]	0	F

Abbreviations: CI = confidence interval; OR = odds ratio; F = fixed-effects mode; R = random-effects model; HB = hospital based; PB = population based.

**Table 3:** Egger's test and Begg's test for publication bias in population.

Genetic comparison	Begg's test (*z*, *p*)	Egger's test (*t*, *p*)
G vs. A	0.21,0.837	-0.53 0.607
GA vs. AA	0.75, 0.451	-0.68, 0.510
GG vs. AA	0.21, 0.837	0.08, 0.940
GA + GG vs. AA	0.62, 0.537	-0.55, 0.593
GG vs. GA + AA	0.07, 0.945	0.16, 0.875

## Data Availability

The data used to support the findings of this study are included within the article.
